# Aberrant Methylation and Differential Expression of SLC2A1, TNS4, GAPDH, ATP8A2, and CASZ1 Are Associated with the Prognosis of Lung Adenocarcinoma

This article has been retracted.

**DOI:** 10.1155/2020/1807089

**Published:** 2020-09-25

**Authors:** Xia Wang, Dongming Shi, Dejun Zhao, Danping Hu

**Affiliations:** Department of Pneumology, The First People's Hospital of Fuyang, Fuyang, China

## Abstract

Lung cancer is one of the leading triggers for cancer death worldwide. In this study, the relationship of the aberrantly methylated and differentially expressed genes in lung adenocarcinoma (LUAD) with cancer prognosis was investigated, and 5 feature genes were identified eventually. Specifically, we firstly downloaded the LUAD-related mRNA expression profile (including 57 normal tissue samples and 464 LUAD tissue samples) and Methy450 expression data (including 32 normal tissue samples and 373 LUAD tissue samples) from the TCGA database. The package “limma” was used to screen differentially expressed genes and aberrantly methylated genes, which were intersected for identifying the hypermethylated downregulated genes (DGs Hyper) and the hypomethylated upregulated genes (UGs Hypo). GO annotation and KEGG pathway enrichment analysis were further performed, and it was found that these DGs Hyper and UGs Hypo were predominantly activated in the biological processes and signaling pathways such as the regulation of vasculature development, DNA-binding transcription activator activity, and Ras signaling pathway, indicating that these genes play a vital role in the initiation and progression of LUAD. Additionally, univariate and multivariate Cox regression analyses were conducted to find the genes significantly associated with LUAD prognosis. Five genes including SLC2A1, TNS4, GAPDH, ATP8A2, and CASZ1 were identified, with the former three highly expressed and the latter two poorly expressed in LUAD, indicating poor prognosis of LUAD patients as judged by survival analysis.

## 1. Introduction

Lung cancer features the second highest incidence (man/woman: 13%) and the top highest mortality (man: 24%, woman: 23%) in the world [1]. It mainly includes small cell lung cancer (SCLC) and non-small cell lung cancer (NSCLC). NSCLC patients account for about 80% of all lung cancer patients. Lung adenocarcinoma (LUAD) is the main histological subtype of NSCLC, accounting for over 40% of all lung cancer cases [2]. About 80% of lung cancer patients are in the advanced stage when they are primarily diagnosed. In this vein, they will lose the optimal operating time, resulting in a very low survival rate and an overall 5-year survival rate only about 17% [3, 4]. Therefore, mining related genes and independent prognostic factors, studying their impact on tumor development and prognosis, and establishing an efficient and stable prognostic model are of great significance for the implementation of precision medicine and the improvement of the cure rate and prognosis of patients.

With the development of tumor-related research, it has been found that genetic variation and epigenetic modification are the two mechanisms that correlate to the occurrence and progression of cancers [5]. DNA methylation is the first discovered epigenetic phenomenon [6]. DNA methylation refers to the transfer of methyl groups to the 5-carbon atom of cytosine in the unmethylated cytosine phosphate guanosine (CpG) dinucleotide under the catalysis of DNA methyltransferase (DNMT) [7, 8], which will result in gene silencing, showing its intimate correlation with the occurrence and development of many diseases [9–12]. Studies have found that abnormal DNA methylation is closely related to the occurrence and development of cancers. In addition, compared with RNA or most protein profiles, the DNA methylation spectrum is more stable and easier to detect. Therefore, many studies have pointed out that DNA methylation-related biomarkers can be used for early diagnosis and prognosis of cancers [13–16]. For instance, Yi and his group [17] discovered that the hypermethylation of BNC1 and ADAMTS1 could be used as biomarkers for the early detection of pancreatic cancer. Additionally, Guo et al. [18] noted that the methylation level of AGTR1, GALR1, SLC5A8, ZMYND10, and NTSR1 is related to the pathogenesis of NSCLC, and the 5 genes could be applied for early diagnosis of NSCLC. Given the abovementioned, we considered that for the early diagnosis and drug development for cancer in the future, it is essential to identify the methylation-related biomarkers that might be involved in LUAD pathogenesis through analysis on the differential methylation in cancer patients.

Evaluation for the early prognosis of patients with lung cancer can improve their survival time and the quality of life. Abnormal DNA methylation usually occurs in the early stage of lung cancer, so it can be used as a potential molecular marker for early prognosis evaluation of lung cancer patients [19]. With the emergence of a large amount of DNA methylation data, researchers can obtain the methylation data of the genes to be studied from free public databases, such as GEO and TCGA databases. A large amount of information in these databases can help researchers find biomarker genes [20]. de Almeida and other colleagues [14] analyzed the DNA methylation and gene expression data between breast cancer tissue and corresponding normal tissue in TCGA and found that cg12374721 (PRAC2), cg18081940 (TDRD10), and cg04475027 (TMEM132C) could be used as diagnostic and prognostic markers in breast cancer. He and other experts [21] analyzed the methylation status of CpG sites and the RNA-seq data of LUAD in TCGA database to explore the relationship regarding the prognostic value between DNA methylation and corresponding gene expression, and then 10 genes were found to be related to the prognosis of patients, indicating that they may be therapeutic targets of LUAD. Although there have been studies on biomarkers for prognosis of LUAD, most of the biomarkers cannot help to accurately predict the prognosis of patients with LUAD. Therefore, it is very important to identify novel prognostic markers to effectively predict the prognosis of patients with LUAD.

In this study, mRNA HTSeq-FPKM-UQ data and Methy450 data related to LUAD were obtained from TCGA database. Then, hypermethylated downregulated genes and hypomethylated upregulated genes were screened, which were sequentially subjected to GO and KEGG enrichment analyses. Furthermore, univariate and multivariate Cox regression analyses were used to screen feature genes significantly related to the prognosis of patients with LUAD. After that, the feasibility of these prognosis-related genes as a prognostic biomarker for patients with LUAD was also verified. These results provide a research basis for improving the prognosis and the life quality of patients with LUAD.

## 2. Materials and Methods

### 2.1. Acquirement of Differentially Expressed Genes and Aberrantly Methylated Genes

HTSeq-FPKM-UQ data of LUAD-related mRNAs were obtained from TCGA database, consisting of 57 normal tissue samples and 464 LUAD tissue samples. R package “limma” was used to perform differential analysis to identify differentially expressed mRNAs, with the normal samples as the control and ∣logFC | >1 along with *P*.adjust < 0.05 as the threshold.

LUAD-related Methy450 data were obtained from TCGA database as well, including 32 normal tissue samples and 373 LUAD tissue samples. The methylation sites with an average beta < 0.01 in all samples were excluded. Similarly, “limma” package was used to screen aberrantly methylated genes (∣logFC | >0.2, *P*.adjust < 0.05). Thereafter, the differentially expressed mRNAs and the aberrantly methylated genes were intersected. The genes which decreased but were highly methylated were defined as the hypermethylated downregulated genes (DGs Hyper), while the genes which increased but were poorly methylated were defined as the hypomethylated upregulated genes (UGs Hypo).

### 2.2. GO Annotation and KEGG Pathway Enrichment Analysis of the DGs Hyper and UGs Hypo

In order to know more about the molecular functions that the DGs Hyper and UGs Hypo play in LUAD, GO annotation and KEGG enrichment analysis were conducted with the aid of the “clusterProfiler” package. GO analysis tends to annotate gene function from three aspects: molecular function, biological process, and cellular components [22–24], while the KEGG pathway enrichment analysis is prone to describe gene function in the genomic and molecular levels and show the correlated genes. *P*.adjust < 0.05 was considered to be statistically significant.

### 2.3. Identification of the Feature Genes Associated with LUAD Prognosis

The DGs Hyper and UGs Hypo were subjected to univariate Cox regression analysis combined with the complete clinical data from the TCGA-LUAD dataset. Genes with *P*.adjust < 0.05 were regarded as the genes correlated to LUAD prognosis. Afterwards, further multivariate Cox regression analysis was performed to identify the feature genes of remarkable prognostic significance.

### 2.4. Verification of the Differential Expression and Aberrant Methylation of the Prognosis-Related Genes

The mRNA data and methylation data from the TCGA-LUAD dataset were used to verify the differential expression and the aberrant methylation of the prognosis-related feature genes.

## 3. Results

### 3.1. Identification of the Differentially Expressed Genes and the Aberrantly Methylated Genes in LUAD

Based on the mRNA expression data and the Methy450 data obtained from the TCGA-LUAD dataset, differential analysis was performed using the R package “limma.” In total, 2,649 differentially expressed mRNAs were obtained (Figure 1(a)), and the screened abnormal methylation sites are listed in Table S1. As revealed, gene expression varied between LUAD cancer tissue and normal tissue. AGER, FAM107A, and GPD1, for instance, were most highly downregulated in cancer tissue, while COL10A1, MMP11, and SPP1 were most significantly upregulated.

Thereafter, the differentially expressed mRNAs and the aberrantly methylated genes were intersected. Eventually, 58 UGs Hypo and 157 DGs Hyper were identified (Figure 1(b)).

### 3.2. GO Annotation and KEGG Pathway Enrichment Analysis of the DGs Hyper and UGs Hypo

To gain more insight into the molecular mechanism of the UGs Hypo and DGs Hyper underlying the initiation and progression of LUAD, GO annotation and KEGG pathway enrichment analysis were carried out using the “clusterProfiler” package. As shown in Figure 2(a), the most enriched GO terms of the total 215 genes were the regulation of vasculature development, DNA-binding transcription activator activity, and RNA polymerase II-specific, while the KEGG analysis revealed that the genes were significantly activated in the signaling pathways involved in human T-cell leukemia virus 1 infection, cell adhesion molecules (CAMs), Ras signaling pathway, and so on (Figure 2(b)). Collectively, the above findings indicate that the UGs Hypo and DGs Hyper might be crucial in the research for the regulatory mechanism of DNA methylation in LUAD.

### 3.3. Identification of Prognosis-Related Genes

To identify the genes associated with LUAD prognosis from the UGs Hypo and DGs Hyper, clinical data of the 474 LUAD patients were obtained from TCGA database for survival analysis. Firstly, the 215 UGs Hypo and DGs Hyper were subjected to univariate Cox regression analysis, and the genes with *P*.adjust < 0.01 were screened and sequentially used for multivariate Cox regression analysis. Eventually, 5 genes were identified to be significantly associated with the prognosis of LUAD, including SLC2A1, TNS4, GAPDH, ATP8A2, and CASZ1 (Figure 3(a)). Survival analysis combined with clinical data revealed that patients with high SLC2A1, TNS4, and GAPDH or low ATP8A2 and CASZ1 had poor prognosis (Figure 3(b)).

### 3.4. Verification of the Differential Expression and the Aberrant Methylation of the Prognosis-Related Genes

Relevant data from the TCGA-LUAD dataset were used to verify the expression and methylation of the prognosis-related genes using the Wilcox test. It turned out that ATP8A2 and CASZ1 were poorly expressed in LUAD tissue, while SLC2A1, TNS4, and GAPDH were highly expressed (Figure 4(a)). Additionally, ATP8A2 and CASZ1 were found to be hypermethylated in tumor samples, and the other three genes were hypomethylated (Figure 4(b)). It could be seen that there was a negative correlation between mRNA expression and methylation. Taken together, we could conclude that the differential expression and the aberrant methylation of SLC2A1, TNS4, GAPDH, ATP8A2, and CASZ1 are significantly associated with the prognosis of LUAD patients.

## 4. Discussion

Increasing studies have found that epigenetic modification exerts a crucial role in the development of LUAD [5, 25, 26]. DNA methylation is a common epigenetic mechanism studied extensively that can regulate gene expression and play an important role in DNA repair, cell adhesion, cell cycle control, and apoptosis regulation [9, 10]. DNA methylation-related biomarkers have also been identified to be used for early diagnosis and prognosis of cancer [15, 27]. A study discovered that the methylation of SHOX2 varies in NSCLC patients at different tumor stages and can be used to judge whether the tumor staging is accurate [28]. Additionally, there was a study on the sputum of lung cancer patients, which successfully identified 4 methylation-related biomarkers, including APC, CDKN2A/p16, HS3ST2 (3OST2), and RASSF1A, and they all can play a part in early screening of lung cancer by serving as biomarkers for early diagnosis [29]. Hence, understanding the mechanism of DNA methylation and exploring the correlation between the differentially expressed genes regulated by abnormal DNA methylation and the prognosis of LUAD patients are of great significance in the improvement of the diagnosis, treatment, and prognosis of LUAD patients.

In this study, DGs Hyper and UGs Hypo were identified. To further understand the role of these genes, we performed GO and KEGG enrichment analyses and discovered that the genes were mainly enriched in biological processes such as the regulation of vasculature development, DNA-binding transcription activator activity, RNA polymerase II-specific, and signaling pathways including the human T-cell virus 1 infection, cell adhesion molecules (CAMs), and Ras signaling pathway. Several studies have reported that vasculature development and DNA-binding transcription activator activity can significantly promote the malignant progression of tumors [30–32]. Cell adhesion molecules are closely related to the invasion and migration of multiple tumors [33–35]. The Ras gene is abnormally expressed in gastric cancer [36], prostate cancer [37], and colorectal cancer [38], and it is associated with epithelial-mesenchymal transition (EMT) and drug resistance of cancer. These evidences suggest that the DGs Hyper and the UGs Hypo may play an important regulatory role in the molecular mechanism of LUAD.

In addition, we also found 5 genes which had differential expression and abnormal methylation in LUAD, including SLC2A1, TNS4, GAPDH, ATP8A2, and CASZ1. Among the 5 genes, ATP8A2 and CASZ1 decreased while SLC2A1, TNS4, and GAPDH increased, which indicated the poor prognosis of patients. The above genes have been found to be abnormally expressed and exert their functions in a variety of cancers. SLC2A1, solute carrier family 2 member 1, can promote glucose uptake by glucose transporters and is able to transport a variety of aldose including pentose and hexose [39–41]. Besides, SLC2A1 is abnormally expressed in various cancers and is associated with cancer proliferation, metastasis, and energy metabolism [42–45]. TNS4 (Tensin 4) is a protein-coding gene that is involved in the cell movement induced by MET and is associated with the GPCR signaling pathway. A study reported that high expression of TNS4 in gastric cancer is associated with poor prognosis [46]. The protein encoded by the ATP8A2 (ATPase Phospholipid Transporting 8A2) gene is a member of the P4 ATPase family of proteins and a catalytic component of the P4-ATPase flippase complex that can catalyze the hydrolysis of ATP involved in the transport of aminophospholipids from the outer to the inner leaflets of diverse membranes and makes sure the phospholipids maintain asymmetrical distribution. It has been noted that ATP8A2 is abnormally methylated in various cancer tissues [47, 48], but its potential molecular mechanism has not been studied. CASZ1 (Castor Zinc Finger 1) encodes a zinc finger transcription factor and has been found to inhibit the growth of neuroblastoma as a tumor suppressor [49–51]. Low expression of CASZ1 is associated with poor prognosis in patients with clear cell renal cell carcinoma [52]. Besides, the hypermethylation of CASZ1 can be used as a biomarker for the diagnosis of esophageal cancinoma [53]. GAPDH (glyceraldehyde-3-phosphate dehydrogenase) has the activities of both glyceraldehyde-3-phosphate dehydrogenase and nitrosylase and functions in glycolysis and nuclear transcription, RNA transport, DNA replication, and apoptosis. It has been found that the high expression of GAPDH is related to the proliferation and invasion of lung cancer and esophageal cancinoma [54], and it can also be used as a serum marker for cervical cancer screening [55]. These studies indicate that SLC2A1, TNS4, GAPDH, ATP8A2, and CASZ1 may participate in the regulation of the occurrence and development of LUAD through DNA methylation and can be used as prognostic markers of LUAD.

Furthermore, assessment for the risk of cancer prognosis based on methylation or gene expression level is common at present. Methylation detection techniques mainly include methylation-specific PCR, bisulfite sequencing, and high-resolution melting (HRM) [56]. Due to the relatively high stability of genomic DNA over mRNA, detection for methylation level can be carried out using blood, sputum, bronchovesicular lavage fluid, and other samples of patients, which are rich and convenient [56]. While for mRNA detection, it has a relatively high demand for samples and transport generally attributed to the liability of mRNA to degrade, indicating less convenience relative to DNA detection. In view of these, this study screened methylation-related biomarkers with prognostic significance in LUAD patients and tended to predict the risk of LUAD prognosis through testing the methylation level of corresponding genes.

In general, the differential expression and the abnormal methylation of SLC2A1, TNS4, GAPDH, ATP8A2, and CASZ1 genes were identified in LUAD patients, and it was found that low expression of ATP8A2 and CASZ1 or high expression of SLC2A1, TNS4, and GAPDH led to poor prognosis of patients. These five genes may play an important role in the DNA methylation mechanism of LUAD, and they may be a promising marker for predicting the prognosis of LUAD patients. Although this study preliminarily discovered that LUAD DNA methylation is related to the prognosis of patients, the specific mechanism is still unclear. Therefore, we will try to further explore the effect of the methylation of these five genes on the occurrence and development of LUAD through cell biological experiments. In addition, this study lacks clinical trials to prove the prognostic genes, and the feasibility of these five genes as prognostic markers in LUAD will be further validated in future clinical trials.

## Figures and Tables

**Figure 1:** Identification of the differentially expressed genes and the aberrantly methylated genes in LUAD. (a) Volcano plot shows the differentially expressed mRNAs in the TCGA-LUAD dataset (red means upregulated genes and blue refers to downregulated genes; green dots are the top 10 downregulated genes in fold change, and purple dots are the top 10 upregulated genes in fold change). (b) Venn diagram is plotted to find the UGs Hypo and DGs Hyper.

**Figure 2:** Functional enrichment analysis of the UGs Hypo and DGs Hyper. (a) The most enriched GO terms for the UGs Hypo and DGs Hyper. (b) The most activated KEGG pathways for the UGs Hypo and DGs Hyper. The dot size represents the number of enriched genes, and the color of the dot represents *P*.adjust (red to green means the *P*.adjust from low to high).

**Figure 3:** Identification of prognosis-related genes. (a) The LUAD prognosis-related genes identified by the multivariate Cox regression analysis. (b) Survival analysis shows the correlation between gene expression (SLC2A1, TNS4, GAPDH, ATP8A2, and CASZ1) and LUAD prognosis.

**Figure 4:** Verification of the differential expression and the aberrant methylation of the prognosis-related genes. (a) The mRNA expression of SLC2A1, TNS4, GAPDH, ATP8A2, and CASZ1 in TCGA-LUAD. (b) The methylation level of SLC2A1, TNS4, GAPDH, ATP8A2, and CASZ1 in TCGA-LUAD.

## Data Availability

The data used to support the findings of this study are included within the article. The data and materials in the current study are available from the corresponding author on reasonable request.

## Supplementary Materials

Supplementary Materials Table S1: The screened abnormal methylation sites.

## References

[1] Siegel R. L., Miller K. D., Jemal A. (2018). Cancer statistics, 2019. *CA: A Cancer Journal for Clinicians*.

[2] Shi J., Hua X., Zhu B. (2016). Somatic genomics and clinical features of lung adenocarcinoma: a retrospective study. *PLoS Medicine*.

[3] Carrato A., Vergnenègre A., Thomas M., McBride K., Medina J., Cruciani G. (2014). Clinical management patterns and treatment outcomes in patients with non-small cell lung cancer (NSCLC) across Europe: EPICLIN-Lung study. *Current Medical Research and Opinion*.

[4] Miller K. D., Siegel R. L., Lin C. C. (2016). Cancer treatment and survivorship statistics, 2016. *CA: a Cancer Journal for Clinicians*.

[5] Wu C., Morris J. R. (2001). Genes, genetics, and epigenetics: a correspondence. *Science*.

[6] Hotchkiss R. D. (1948). The quantitative separation of purines, pyrimidines, and nucleosides by paper chromatography. *The Journal of Biological Chemistry*.

[7] Morgan A. E., Davies T. J., Mc Auley M. T. (2018). The role of DNA methylation in ageing and cancer. *The Proceedings of the Nutrition Society*.

[8] Holčáková J. (2018). Effect of DNA methylation on the development of cancer. *Klinicka Onkologie: Casopis Ceske a Slovenske Onkologicke Spolecnosti*.

[9] Guo H., Zhu P., Yan L. (2014). The DNA methylation landscape of human early embryos. *Nature*.

[10] Huo Z., Zhu Y., Yu L. (2019). DNA methylation variability in Alzheimer’s disease. *Neurobiology of Aging*.

[11] Zinellu A., Sotgiu E., Fois A. G. (2017). Blood global DNA methylation is decreased in non-severe chronic obstructive pulmonary disease (COPD) patients. *Pulmonary Pharmacology & Therapeutics*.

[12] Kommoss F. K. F., Stichel D., Schrimpf D. (2020). DNA methylation-based profiling of uterine neoplasms: a novel tool to improve gynecologic cancer diagnostics. *Journal of Cancer Research and Clinical Oncology*.

[13] Mathios D., Hwang T., Xia Y. (2019). Genome-wide investigation of intragenic DNA methylation identifies ZMIZ1 gene as a prognostic marker in glioblastoma and multiple cancer types. *International Journal of Cancer*.

[14] de Almeida B. P., Apolónio J. D., Binnie A., Castelo-Branco P. (2019). Roadmap of DNA methylation in breast cancer identifies novel prognostic biomarkers. *BMC Cancer*.

[15] Hu W. L., Zhou X. H. (2017). Identification of prognostic signature in cancer based on DNA methylation interaction network. *BMC Medical Genomics*.

[16] Zan Y., Wang B., Liang L. (2019). MicroRNA-139 inhibits hepatocellular carcinoma cell growth through down-regulating karyopherin alpha 2. *Journal of Experimental & Clinical Cancer Research*.

[17] Yi J. M., Guzzetta A. A., Bailey V. J. (2013). Novel methylation biomarker panel for the early detection of pancreatic cancer. *Clinical Cancer Research*.

[18] Guo S., Yan F., Xu J. (2015). Identification and validation of the methylation biomarkers of non-small cell lung cancer (NSCLC). *Clinical Epigenetics*.

[19] Johnson L., Mercer K., Greenbaum D. (2001). Somatic activation of the K-ras oncogene causes early onset lung cancer in mice. *Nature*.

[20] Gao C., Zhou C., Zhuang J. (2018). MicroRNA expression in cervical cancer: novel diagnostic and prognostic biomarkers. *Journal of Cellular Biochemistry*.

[21] He W., Ju D., Jie Z., Zhang A., Xing X., Yang Q. (2018). Aberrant CpG-methylation affects genes expression predicting survival in lung adenocarcinoma. *Cancer Medicine*.

[22] Mazandu G. K., Chimusa E. R., Mulder N. J. (2016). Gene Ontology semantic similarity tools: survey on features and challenges for biological knowledge discovery. *Briefings in Bioinformatics*.

[23] Meijer R. J., Goeman J. J. (2016). Multiple testing of gene sets from Gene Ontology: possibilities and pitfalls. *Briefings in Bioinformatics*.

[24] Zhang C., Zheng W., Freddolino P. L., Zhang Y. (2018). MetaGO: predicting Gene Ontology of non-homologous proteins through low-resolution protein structure prediction and protein-protein network mapping. *Journal of Molecular Biology*.

[25] Wang Y., Deng H., Xin S., Zhang K., Shi R., Bao X. (2019). Prognostic and predictive value of three DNA methylation signatures in lung adenocarcinoma. *Frontiers in Genetics*.

[26] Li H., Tong L., Tao H., Liu Z. (2020). Genome-wide analysis of the hypoxia-related DNA methylation-driven genes in lung adenocarcinoma progression. *Bioscience Reports*.

[27] Li P., Liu J., Li J., Liu P. (2019). DNA methylation of CRB3 is a prognostic biomarker in clear cell renal cell carcinoma. *Molecular Biology Reports*.

[28] Kneip C., Schmidt B., Seegebarth A. (2011). SHOX2 DNA methylation is a biomarker for the diagnosis of lung cancer in plasma. *Journal of Thoracic Oncology*.

[29] Shivapurkar N., Stastny V., Suzuki M. (2007). Application of a methylation gene panel by quantitative PCR for lung cancers. *Cancer Letters*.

[30] Minder P., Zajac E., Quigley J. P., Deryugina E. I. (2015). EGFR regulates the development and microarchitecture of intratumoral angiogenic vasculature capable of sustaining cancer cell intravasation. *Neoplasia*.

[31] Brown H. M., Russell D. L. (2014). Blood and lymphatic vasculature in the ovary: development, function and disease. *Human Reproduction Update*.

[32] Aggarwal B. B., Kunnumakkara A. B., Harikumar K. B. (2009). Signal transducer and activator of transcription-3, inflammation, and cancer: how intimate is the relationship?. *Annals of the New York Academy of Sciences*.

[33] Pisamai S., Rungsipipat A., Kalpravidh C., Suriyaphol G. (2017). Gene expression profiles of cell adhesion molecules, matrix metalloproteinases and their tissue inhibitors in canine oral tumors. *Research in Veterinary Science*.

[34] Lian S., Lu Y., Cheng Y. (2016). S-Nitrosocaptopril interrupts adhesion of cancer cells to vascular endothelium by suppressing cell adhesion molecules via inhibition of the NF-кB and JAK/STAT signal pathways in endothelial cells. *European Journal of Pharmacology*.

[35] Zheng J., Hernandez J. M., Doussot A. (2018). Extracellular matrix proteins and carcinoembryonic antigen-related cell adhesion molecules characterize pancreatic duct fluid exosomes in patients with pancreatic cancer. *HPB: The Official Journal of the International Hepato Pancreato Biliary Association*.

[36] Ge P., Wei L., Zhang M. (2018). TRPC1/3/6 inhibition attenuates the TGF-*β*1-induced epithelial-mesenchymal transition in gastric cancer via the Ras/Raf1/ERK signaling pathway. *Cell Biology International*.

[37] Huang L., Wang L., Wang L. (2020). MicroRNA let-7b inhibits proliferation and induces apoptosis of castration-resistant prostate cancer cells by blocking the Ras/rho signaling pathway via NRAS. *Clinical and Translational Science*.

[38] Zhang X., Liu G., Ding L. (2018). HOXA3 promotes tumor growth of human colon cancer through activating EGFR/Ras/Raf/MEK/ERK signaling pathway. *Journal of Cellular Biochemistry*.

[39] Mueckler M., Makepeace C. (2008). Transmembrane segment 6 of the Glut1 glucose transporter is an outer helix and contains amino acid side chains essential for transport activity. *The Journal of Biological Chemistry*.

[40] Mueckler M., Makepeace C. (2009). Model of the exofacial substrate-binding site and helical folding of the human Glut1 glucose transporter based on scanning mutagenesis. *Biochemistry*.

[41] Lee E. E., Ma J., Sacharidou A. (2015). A protein kinase C phosphorylation motif in GLUT1 affects glucose transport and is mutated in GLUT1 deficiency syndrome. *Molecular Cell*.

[42] Ding X., Liu J., Liu T., Ma Z., Wen D., Zhu J. (2017). miR-148b inhibits glycolysis in gastric cancer through targeting SLC2A1. *Cancer Medicine*.

[43] Santasusagna S., Moreno I., Navarro A. (2018). miR-328 mediates a metabolic shift in colon cancer cells by targeting SLC2A1/GLUT1. *Clinical & translational oncology: official publication of the Federation of Spanish Oncology Societies and of the National Cancer Institute of Mexico*.

[44] Yan S., Wang Y., Chen M., Li G., Fan J. (2015). Deregulated SLC2A1 promotes tumor cell proliferation and metastasis in gastric cancer. *International Journal of Molecular Sciences*.

[45] Ooi A. T., Gomperts B. N. (2015). Molecular pathways: targeting cellular energy metabolism in cancer via inhibition of SLC2A1 and LDHA. *Clinical Cancer Research: An Official Journal of the American Association for Cancer Research*.

[46] Sakashita K., Mimori K., Tanaka F. (2008). Prognostic relevance of Tensin4 expression in human gastric cancer. *Annals of Surgical Oncology*.

[47] Yan H., Guan Q., He J. (2017). Individualized analysis reveals CpG sites with methylation aberrations in almost all lung adenocarcinoma tissues. *Journal of Translational Medicine*.

[48] Ohara K., Arai E., Takahashi Y. (2017). Genes involved in development and differentiation are commonly methylated in cancers derived from multiple organs: a single-institutional methylome analysis using 1007 tissue specimens. *Carcinogenesis*.

[49] Liu Z., Yang X., Li Z. (2011). CASZ1, a candidate tumor-suppressor gene, suppresses neuroblastoma tumor growth through reprogramming gene expression. *Cell Death and Differentiation*.

[50] Wang C., Liu Z., Woo C. W. (2012). EZH2 mediates epigenetic silencing of neuroblastoma suppressor genes CASZ1, CLU, RUNX3, and NGFR. *Cancer Research*.

[51] Liu Z., Naranjo A., Thiele C. J. (2011). CASZ1b, the short isoform of CASZ1 gene, coexpresses with CASZ1a during neurogenesis and suppresses neuroblastoma cell growth. *PLoS One*.

[52] Kim B., Jung M., Moon K. C. (2019). The prognostic significance of protein expression of CASZ1 in clear cell renal cell carcinoma. *Disease Markers*.

[53] Wang H. Q., Yang C. Y., Wang S. Y. (2018). Cell-free plasma hypermethylated CASZ1, CDH13 and ING2 are promising biomarkers of esophageal cancer. *Journal of Biomedical Research*.

[54] Hao L., Zhou X., Liu S. (2015). Elevated GAPDH expression is associated with the proliferation and invasion of lung and esophageal squamous cell carcinomas. *Proteomics*.

[55] Xu M. L., Kim H. J., Kim S. C. (2019). Serum anti-GAPDH autoantibody levels reflect the severity of cervical lesions: a potential serum biomarker for cervical cancer screening. *Oncology Letters*.

[56] Anglim P. P., Alonzo T. A., Laird-Offringa I. A. (2008). DNA methylation-based biomarkers for early detection of non-small cell lung cancer: an update. *Molecular Cancer*.

